# Information Monitoring of Animal Husbandry Industry Based on the Internet of Things and Wireless Communication System

**DOI:** 10.1155/2022/8794044

**Published:** 2022-03-28

**Authors:** Yuhong Shen

**Affiliations:** Physics and Electronic Information College, Hulunbuir University, Hulunbuir, 021008 Inner Mongolia, China

## Abstract

This paper was aimed at discussing the information monitoring of animal husbandry based on the Internet of Things and wireless communication system. The breeding and health of animals in the breeding industry has always been a topic that people talk about. The advent of the wireless communication system has made monitoring and positioning technologies more and more simple. The wireless communication network technology is applied to the environmental monitoring of animal breeding farms, and a real-time reporting system is designed to pay attention to animal health in real time. This article focuses on the connection between the two. First, this article briefly describes the state of the wireless communication network and the aquaculture industry, furthermore explains the research methods, such as the livestock breeding environment monitoring system model, which needs to have the characteristics of humanization, fast and simple, easy to maintain, high reliability, compatibility, scalability, and intelligence, and designs related monitoring systems and hardware systems to integrate carbon dioxide, ammonia, and other gas sensors with temperature and humidity sensors to sense the environment. Next, this article shows the wireless communication network monitoring and positioning algorithm, namely, the TOA-based wireless communication positioning algorithm and the LTE prediction algorithm. The predicted time is used as the link weight, and the weight within the wide link cluster is defined according to the time threshold, making the link maintain stability for a short time to enhance the network topology. Then, this article conducts experiments based on ZigBee wireless communication network sensor combined with improved genetic algorithm in the temperature and humidity test of farms, designs the environmental monitoring system, improves the algorithm, and cooperates with experiments and analysis to verify the feasibility and apply it to the temperature and humidity test of the livestock farm. The results are good, and the temperature and humidity errors are reduced by 88.28% and 84.21%, respectively. It has a certain degree of guidance. Finally, it is discussed and summarized. It can be seen that the system and algorithm designed in this paper have a good prospect in the development of animal husbandry. However, this algorithm takes a long time and has a broader research space.

## 1. Introduction

The economic situation in the society is constantly improving, so people's requirements for living standards are also constantly improving, and the demand for fresh meat food is rising day by day. In such an environment, people's requirements for food quality will be more stringent, safe and harmless, green and pollution-free, etc., which has become one of the criteria for judging the quality of food. Therefore, the country's requirements for the breeding industry are even more stringent, especially the emergence of unfavorable infectious diseases such as avian influenza and mad cow disease, which necessitates changes and improvements in the prior breeding technology. The use of new breeds and detection and monitoring technologies can adapt to the needs of the general environment. This article focuses on the breeding situation of animals in livestock houses and conducts targeted research and exploration in terms of breeding process, breeding environment, breeding monitoring, etc., and establishes a low-cost, high-stability livestock breeding environment monitoring system suitable for the breeding industry. Livestock breeding has gradually been industrialized, diversified, and integrated, but the breeding environment is still a major problem hindering the development of the breeding industry. Therefore, farmers should focus on calibrating the standards of the breeding environment. The breeding environment has a greater impact on the stable growth of livestock, and summer and winter are very unfavorable for livestock production, resulting in a decrease in livestock production capacity by about 10% to 20%. At the same time, high temperature and cold will also have a great impact on the health and development of livestock. Therefore, timely and effective monitoring of the quality of the breeding environment can reduce the impact of the environment on livestock to a reasonable range. The temperature and humidity in the breeding environment, gas concentration, light intensity and intensity, etc., will all have varying degrees of impact on the development and reproduction of livestock, and it is necessary to arrange corresponding sensors. It is necessary to analyze and establish the breeding environment in advance. According to the environmental characteristics, it is necessary to arrange suitable monitoring facilities and systems, so as to monitor the harmful components in the breeding environment in real time and provide powerful reference data for subsequent treatment and improvement.

ZigBee communication networking technology has been widely used in various fields, especially in the field of low speed; it has been widely used in M2M industries in the IoT industry chain, such as smart grid, smart transportation, smart home, finance, mobile POS terminals, supply chain automation, industrial automation, smart buildings, fire protection, public safety, environmental protection, meteorology, digitalization Medical, telemetry, agriculture, forestry, water, coal, petrochemical, and other fields [1, 2]. In the short-distance wireless personal local area networks, the emergence of this technology has played a vital role in the establishment of a breeding environment monitoring system. Whether it is data transmission or remote control and viewing, it needs to be developed and designed based on ZigBee technology. Through this technology, a high proportion of automatic operations can be realized, such as automatic transmission and processing of data and automatic generation of data curve graphics, and remote control and viewing functions of users can also be realized. Under the guidance of this technology, various troubles caused by complicated on-site wiring and postmaintenance are avoided. The construction cost and maintenance cost of traditional breeding environment detection technology are much higher than this technology. Not only that ZigBee technology is far superior to traditional detection technology in terms of data acquisition accuracy, sensitivity, and transmission performance. While bringing convenience to users, it also brings obvious advantages of low cost and high experience. This technology can provide stable and reliable technical support for monitoring and control and improve the current breeding management mode and has great significance in terms of breeding safety, quality, and safety.

This article uses ZigBee communication networking technology to design an environmental monitoring system that can monitor temperature, humidity, NH3 concentration, etc., combined with the proposed algorithm based on traditional genetic algorithms, mutation operators, and hybrid operators to improve the temperature in the farm, using humidity sensor test experiment. Finally, it is concluded that there are better results, small errors, stable performance, and strong guidance.

## 2. Related Work

Wireless network communication technology has research significance in various fields. Yuan et al. studied the approximate traversal secrecy rate of the two beamformers of the relay: (1) generalized matched forwarding (GMF) beamformer to maximize the legal channel rate and (2) general rank beamformer (GRBF). In addition, a lower limit maximization (LBM) beamformer at the relay is also discussed, which is used to maximize the lower limit of the traversal secrecy [3]. Yao et al. considers a cluster-based cooperative spectrum sensing (CSS) scheme in the Energy Harvesting Cognitive Wireless Communication Network (EH-CWCN), in which cognitive nodes (CN) are clustered according to their received power levels to improve sensing performance. In the CSS scheme, time resources are limited and shared by energy harvesting, spectrum sensing, and data transmission [4]. Jee et al. said that there are more than 300 standard blocks defined in the IEC61131-3 standard, but the existing mutation operator set does not fully cover the functional elements of the FBD program. And by comprehensively considering the functional elements that can be used in the FBD program and the types of errors that may appear in the FBD program, additional mutation operators are defined and through a case study to evaluate the impact of mutation operator expansion [5]. Zhang and Ming believes that its application is limited due to its imperfect search structure and the risk of falling into a local optimum. In order to improve the performance of the algorithm, an optimized GWO (MR-GWO) based on mutation operator and elimination reconstruction mechanism is proposed. The introduction of mutation operator facilitates better search, and the elimination-reconstruction mechanism is adopted for the search of the difference, which not only effectively expands the random search but also accelerates its convergence [6]. Friggens et al. said that as the environment for raising livestock becomes more and more variable, the robustness of animals has become an increasingly valuable attribute. Therefore, people pay more and more attention to its management and cultivation. However, robustness is a phenotype that is difficult to correctly characterize because it is a complex feature consisting of multiple components, including dynamic elements, such as response rate and recovery rate to environmental disturbances [7]. In view of the current situation of green environmental protection lighting policy and the problems of high automation, low energy efficiency, and difficult management of traditional residential lighting systems, Liang and Xu proposed a residential community street lamp monitoring and management system based on ZigBee and GPRS. This design is proposed using sensor technology, ZigBee, and GPRS wireless communication technology network. In order to realize intelligent lighting parameter adjustment, a coordinated control method of multiple sensors is adopted [8]. These studies have a certain degree of guidance, but there are insufficient arguments or insufficient precision, which can be further improved.

## 3. Livestock House Monitoring Model and Wireless Communication Network Algorithm

### 3.1. Model of Monitoring System for Livestock Breeding Environment

The design and realization of the whole system should be changed according to the actual situation. The layout of the various sensors in the entire system also needs to be adapted to local conditions and cannot cause cumbersome and interference [9, 10]. Therefore, the overall system design needs to be carried out in accordance with the following rules:

1. Humanization of operation: the whole system highlights the intelligent mode of human-computer interaction. It is not only necessary to pay attention to the richness of system functions but also to consider whether the various functions will cause operational problems for farmers and workers. The main interface of the system should display the frequently used functions and operation buttons, which can be reached directly by one key without repeated operations. At the same time, efforts should be made to reduce the operational interference items in the software design to prevent the adverse consequences caused by misoperation [11]
2. Fast and simple: the operation of the various sensing lines in the system can be adjusted quickly, while providing users with a higher degree of freedom of independent customization functions. The system must not only preset a certain amount of practical parameters but also provide users with space for independent adjustment. And in the interface of the data report of the sensor, the displayed data strives to be simple and direct [12]
3. Easy to maintain and high reliability: because the user groups of the system are generally farmers and workers, all require both software and hardware to maintain good stability under long-term working conditions. At the same time, the reserved software and hardware maintenance interface should also be easy to view. The data acquisition equipment of the sensor needs to have the function of directly displaying the data in order to read and analyze the data intuitively [13]
4. Compatible scalability: as mentioned above, when designing software and hardware, it is necessary to reserve interfaces for subsequent maintenance. These interfaces also have to undertake upgrades and extensions to reduce the user's expenditure in subsequent use. The entire system should achieve dual compatibility and stable use of software and hardware for various equipment and new equipment to be implemented in the future. In this way, the entire system can maintain a long use cycle without causing waste of resources [14]
5. Intelligence: in the current technological environment, artificial intelligence is a big craze. In terms of software functions, it is necessary to intelligently recognize and correct errors and eliminate risks for users in a timely manner. At the same time, prompt and notify in a conspicuous position to improve work efficiency [15]

The livestock breeding environment monitoring system is designed based on a variety of existing mature technologies, such as database technology, remote communication technology, sensor technology, and computer technology. Therefore, from an overall perspective, the entire system has the characteristics of complexity and comprehensiveness. The whole system consists of three parts, namely, environmental monitoring communication networking equipment, data collection system, and remote reading system. The data collection system has functional modules such as visual report definition, audit relationship definition, report approval and release, data reporting, data preprocessing, data review, and comprehensive query statistics. The specific framework is shown in Figure 1.

The environmental monitoring communication networking equipment is composed of a variety of sensors and network equipment. Among them, the sensors include temperature and humidity detection, light intensity detection, and gas concentration detection, and the network equipment is mainly based on ZigBee networking equipment, GRPS wireless communication, and RS485-wired communication equipment [16, 17]. Therefore, the entire system has both wired communication and wireless communication functions, which can be operated on the spot, and can also be controlled remotely, which enriches the user's choice space. The remote reading system is mainly able to provide users with mobile terminal query and control functions, including sensor data query, overall data curve query, and remote control of related hardware devices [18]. The data collection system mainly provides operations such as data collection, processing, and uploading and at the same time receives remote instructions from the user's mobile terminal [19].

The normal operation of the software is based on hardware. Therefore, the hardware system is the physical basis of the entire livestock breeding environment monitoring system. When the hardware system meets the conditions, we can optimize more physical devices, such as display screens and communication antennas. The hardware system includes environmental monitoring and communication networking equipment. The responsibility of these equipment is to detect the data in the environment and transmit it to the cloud in real time [20]. Environmental monitoring and communication networking are interdependent, and the data provided by environmental monitoring equipment needs to be transmitted and stored to the data collection system through the communication networking equipment.  Figure 2 shows the overall structure of the hardware system.

In the entire livestock breeding environment, the space occupied by the equipment is optimized, and the carbon dioxide, ammonia, and other gas sensors and the temperature and humidity sensors are integrated on a panel, which is called the parameter sensing concentrator in the breeding environment [21]. The device has both networking and wired interfaces, namely, RS485 and ZigBee, which is convenient for data upload. At the same time, the equipment is equipped with an LCD display screen and supports keyboard operation, which is convenient for real-time on-site query and analysis of environmental data. The concentrator effectively reduces the environmental space occupied by multisensor laying and realizes multifunctional integration under the small-sized precursor [22]. Therefore, the device cannot only be fixed in a certain environment for use, but its high degree of integration makes it easy to carry. The overall structure of the environmental parameter sensing concentrator is shown in Figure 3.

### 3.2. Wireless Communication Network Monitoring and Positioning Algorithm

#### 3.2.1. TOA-Based Wireless Communication Positioning Algorithm

When there are more than 3 wireless network node distance measurement values, the corresponding two-dimensional estimation result will be obtained. At this time, a set of nonlinear equations will be formed. The solution to this equation is the exact positioning point. This equation is obtained by combining the distance equations of the node and the mobile terminal in the LOS environment. The trilateral algorithm in this problem is shown in Figure 4.

This problem can be solved by the maximum likelihood method and the least square method. In the maximum likelihood method, the optimal estimation value must satisfy the maximum condition probability density function. Letting $\hat{\phi }={\left[\overset{\wedge }{a},\overset{\wedge }{b}\right]}^{n}$ be the estimated coordinates and *ϕ* = [*a*, *b*]^*n*^ be the real coordinates, *n* in the estimated coordinates is the bias factor. Letting $\hat{w}=w+s$ be the ranging vector of the wireless communication base station and *s* be the zero mean Gaussian noise and be in the independent and identically distributed state, then the conditional probability *p* can be obtained as

(1) $$\begin{array}{c} \hat{\phi }=\arg\underset{\phi }{\max}p\left(\hat{w}\left|\phi \right.\right),\\ p\left(\hat{w}\left|\phi \right.\right)=\overset{M}{\underset{k=1}{\prod }}\frac{1}{\sqrt{2{\pi \sigma }_{k}^{2}}}\exp\left\{-\frac{{\left({\overset{\wedge }{w}}_{k}-w_{k}\right)}^{2}}{2\sigma_{k}^{2}}\right\}. \end{array}$$

In this formula, *σ*_*k*_^2^ is the variance of the *k* ranging noise. At this time, the approximate maximum likelihood algorithm is used to solve the problem that cannot be solved in the maximum likelihood method. The approximate likelihood method used is a two-step ML (TS-ML) algorithm. There are also linear least squares and nonlinear least squares based on TOA data, letting *λ*_*ef*_(*ϕ*) be the prediction result and the difference measurement between Euclidean distance ‖*ϕ* − *ϕ*_*k*_‖ and distance measurement ${\hat{w}}_{k}$ between wireless communication base stations. *μ*_*k*_ is one of the weighted values, which can adjust the weight of the equation. The algorithm can obtain the weight value based on the variance value of the node data and other data, and then, the positioning estimation algorithm of the nonlinear algorithm is

(2) $$\begin{array}{c} \hat{\phi }=\arg\underset{\phi }{\min}\left\{\lambda_{ef}\left(\phi \right)\right\}=\arg\underset{\phi }{\min}\left\{\overset{m}{\underset{k=1}{\sum }}\mu_{k}\left({\hat{w}}_{k}-\left\|\phi -\phi_{k}\right\|\right)\left.{}^{2}\right)\right\}. \end{array}$$

The linear least squares rule is to linearize a nonlinear equation:

(3) $$\begin{array}{c} G\left(\phi \right)=\left[\begin{array}{c} \sqrt{{\left(a-a_{1}\right)}^{2}+{\left(b-b_{1}\right)}^{2}},\\ \sqrt{{\left(a-a_{2}\right)}^{2}+{\left(b-b_{2}\right)}^{2}},\\ \vdots \\ \sqrt{{\left(a-a_{M}\right)}^{2}+{\left(b-b_{M}\right)}^{2}}. \end{array}\right] \end{array}$$

The coordinate of base station *m* is [*x*_*m*_, *y*_*m*_], and it is expanded at position *ϕ*_0_ through Taylor expansion. There is *G*(*ϕ*) ≈ *G*(*ϕ*_0_) + *Q*(*ϕ* − *ϕ*_0_), and *Q*(*ϕ* − *ϕ*_0_) are the Jacobian matrix with *Q* at position *ϕ*_0_, and we can get

(4) $$\begin{array}{c} Q={\left[\begin{array}{cccc} \frac{\partial g_{1}}{\partial a} & \frac{\partial g_{2}}{\partial a} & \cdots & \frac{\partial g_{m}}{\partial a}\\ \frac{\partial g_{1}}{\partial b} & \frac{\partial g_{2}}{\partial b} & \cdots & \frac{\partial g_{m}}{\partial b} \end{array}\right]}_{\phi =\phi_{0}}^{N}. \end{array}$$

At this time, the solution of the linear least squares can be solved as

(5) $$\begin{array}{c} \hat{\phi }=\phi_{0}+{\left(Q^{H}Q\right)}^{-1}Q^{H}\left[\hat{w}-G\left(\phi_{0}\right)\right], \end{array}$$

where *H* represents the Hermitian transposition and the lower bound of the Krameruo offline prediction variance using the LLS positioning algorithm:

(6) $$\begin{array}{c} E\left[{\left(\overset{\wedge }{\phi }-\phi \right)}^{2}\right]\geq {Ι}^{-1}\left(\phi \right). \end{array}$$

*E*(•) is the expected value, and I(*φ*) is the Fisher information matrix; we can get

(7) $$\begin{array}{c} I\left(\varphi \right)\overset{\Delta }{=}E\left[{\left(\frac{\partial }{\partial \varphi }1\text{n }g\left(\overset{\wedge }{w}\left|\varphi \right.\right)\right)}^{2}\right]=E\left[\frac{\partial }{\partial \varphi }1\text{n }g\left(\hat{w}\left|\varphi \right.\right).{\left(\frac{\partial }{\partial \varphi }1\text{n }g\left(\overset{\wedge }{w}\left|\varphi \right.\right)\right)}^{N}\right]. \end{array}$$

In formula (7), $g\left(\hat{w}\left|\phi \right.\right)$ is the joint PDF of $\hat{w}$; letting $\hat{w}=w+s$ be the true distance between the wireless communication base station and the MS, *s* is the zero mean Gaussian noise, and *w* is a function of *ϕ*, because

(8) $$\begin{array}{c} \frac{\partial }{\partial \phi }\ln g\left(\hat{w}\left|\phi \right.\right)=\frac{\partial w}{\partial \phi }\cdot \frac{\partial }{\partial w}\ln g\left(\hat{w}\left|w\right.\right). \end{array}$$

So,

(9) $$\begin{array}{c} \begin{array}{c} I\left(\phi \right)=E\left[\frac{\partial }{\partial \phi }\ln g\left(\hat{w}\left|\phi \right.\right)\cdot {\left(\frac{\partial }{\partial \phi }\ln g\left(\overset{\wedge }{w}\left|\phi \right.\right)\right)}^{N}\right]=\\ \frac{\partial w}{\partial \phi }E\left[\frac{\partial }{\partial \phi }\ln g\left(\hat{w}\left|\phi \right.\right)\cdot {\left(\frac{\partial }{\partial \phi }\ln g\left(\overset{\wedge }{w}\left|\phi \right.\right)\right)}^{N}\right]{\frac{\partial w}{\partial \phi }}^{N},\;I\left(\phi \right)=Q{Ι}_{w}Q^{N}, \end{array} \end{array}$$

where *Q* is

(10) $$\begin{array}{c} Q=\left[\begin{array}{ccc} \frac{a-a_{1}}{\sqrt{{\left(a-a_{1}\right)}^{2}+{\left(b-b_{1}\right)}^{2}}} & \cdots & \frac{a-a_{M}}{\sqrt{{\left(a-a_{N}\right)}^{2}+{\left(b-b_{M}\right)}^{2}}}\\ \frac{b-b_{1}}{\sqrt{{\left(a-a_{1}\right)}^{2}+{\left(b-b_{1}\right)}^{2}}} & \cdots & \frac{b-b_{M}}{\sqrt{{\left(a-a_{N}\right)}^{2}+{\left(b-b_{M}\right)}^{2}}} \end{array}\right],\\ I_{w}=\Sigma^{-1}=\mathrm{diag}\left(\sigma_{1}^{-2},\sigma_{1}^{-2},\cdots ,\sigma_{M}^{-2}\right). \end{array}$$

It can get the CRLB of MS position estimation:

(11) $$\begin{array}{c} I{\left(\phi \right)}^{-1}={\left(Q{Ι}_{w}Q^{N}\right)}^{-1}. \end{array}$$

#### 3.2.2. LTE Prediction Algorithm

This algorithm uses an effective link time prediction algorithm to stabilize the network state; the actual link survival time value and the estimated time value can be estimated under the condition that the error formed is not large.  Figure 5 is a simplified time estimation model to simplify the complex calculation data.

Taking the coordinates of the rectangular coordinate system as the model vector, then use the vector to get the correlation quantity. At this time, the coordinate of *m* is *S*_*m*_ = (*x*_*m*_, *y*_*m*_), and the coordinate of *n* is *S*_*n*_ = (*x*_*n*_, *y*_*n*_), and the initial speed is *v*_*mo*_ and, and the acceleration is *a*_*mo*_ and *a*_*no*_. The target rates are *v*_*mp*_ and *v*_*np*_, and the model directions are *μ*and *ω*. The specific calculation process of LTE is as follows:

(i) Step 1: the initial rate and *v*_*no*_ target rate of nodes *m* and *n* are as follows:
  (12) $$\begin{array}{c} v_{mo}=\left(v_{mo}\sin\mu ,v_{mo}\cos\mu \right)\\ v_{mp}=\left(v_{mp}\sin\mu ,v_{mp}\cos\mu \right)\\ v_{no}=\left(v_{no}\sin\omega ,v_{no}\cos\omega \right)\\ v_{np}=\left(v_{np}\sin\omega ,v_{np}\cos\omega \right) \end{array}$$
(ii) Step 2: the initial relative speed *v*_*o*_ and target relative speed *v*_*p*_between nodes *m* and *n* are as follows:
  (13) $$\begin{array}{c} v_{o}=v_{mo}-v_{no}=\left(v_{mo}\sin\mu -v_{no}\sin\omega ,v_{mo}\cos\mu -v_{no}\cos\omega \right)\\ v_{p}=v_{mp}-v_{np}=\left(v_{mp}\sin\mu -v_{np}\sin\omega ,v_{mp}\cos\mu -v_{np}\cos\omega \right) \end{array}$$
(iii) Step 3: calculating the relative position *S* and distance *d* between nodes *m* and *n*:
  (14) $$\begin{array}{c} S=S_{n}-S_{m}=\left(x_{n}-x_{m},y_{n}-y_{m}\right),d=\left|S\right| \end{array}$$

In this formula, *x*_*m*_ and *y*_*m*_, respectively, refer to the size of the abscissa and ordinate of the node *m*, and similarly, *x*_*n*_ and *y*_*n*_, respectively, refer to the size of the abscissa and ordinate of the node *n*

(iv) Step 4: obtaining the required movement distance *h* and relative acceleration *a*′ outside the included angle *ϕ* and the communication range *k* between nodes *m* and *n* through the above formula:
  (15) $$\begin{array}{c} v_{o}\cdot S=\left|v_{o}\right|\left|S\right|\cos\phi \\ h^{2}+d^{2}-2hd\cos\phi =k^{2}\\ a^{\prime }=\left|a_{m}-a_{n}\right| \end{array}$$

In this formula, *a*_*m*_ and *a*_*n*_, respectively, represent the acceleration of each node and its neighboring nodes

(v) Step 5: solving the time required for the node from the initial relative speed to the final relative speed *t*_*o*_ and the travel distance of the acceleration phase *l*_*o*_:
  (16) $$\begin{array}{c} t_{o}=\frac{v_{p}-v_{o}}{\hat{a}};l_{o}=\frac{v_{p}^{2}-v_{o}^{2}}{2\hat{a}} \end{array}$$
(vi) Step 6: determining whether the movement distance of the acceleration stage is smaller than the movement distance, make the node perform a uniform linear movement, let *t*_2_ be the node acceleration time, and solve the link survival time *LTE*(*m*, *n*):
  (17) $$\begin{array}{c} l_{o}+v_{p}t_{1}=h;LET\left(m,n\right)=t_{o}+t_{1}\\ v_{o}t_{2}+\frac{1}{2}\hat{a}{t_{2}}^{2}=h;LET\left(m,n\right)=t_{2} \end{array}$$

1The link survival time is solved. The predicted time is used as the link weight, and the weight in the wide link cluster is defined according to the time threshold. Promoting the link will not be disconnected for a short time, maintain continuous stability, thereby enhancing the network topology

## 4. Experiments Based on ZigBee Wireless Communication Network Sensor Combined with Improved Genetic Algorithm in the Temperature and Humidity Test of Farms

### 4.1. Design of a Farm Information Monitoring System Based on ZigBee Wireless Communication Network Sensors

The information collection subsystem in the breeding environment is mainly composed of three nodes, which are sensor detection nodes, router nodes, and coordinator nodes. The coordinated work of the three has enabled the ZigBee wireless communication technology with CC2530 as the core to successfully collect data in the breeding environment [23]. Among the three nodes, the sensor detection node is mainly responsible for collecting real-time data of various sensors in the breeding environment, such as temperature and humidity, gas concentration, and water and electricity consumption. The layout of sensor detection nodes requires a reasonable analysis of the breeding environment. Through the data collection of all sensor detection nodes in the breeding environment, after calculation by the ZigBee sensor node, the data is converted into data frames and transmitted. The entire transmission process needs to rely on the router node, which provides the wireless forwarding function for the transportation process. The data from the ZigBee sensor node is transmitted through the router node and sent to the final coordinator node. The coordinator node has the highest authority in the entire system. It has the authority to determine the joining and leaving of each node, and it can also receive the incoming data from each node. After all the data is summarized at the coordinator node, it is finally transmitted to the corresponding monitoring system. The subsystem of the monitoring system of the entire host computer is responsible for the data collection and monitoring of the entire ZigBee network system. The host computer monitoring system is designed using Delphi technology. By combining the database of SQL Server2005 to store sensor data, it connects the coordinator node in the information collection system and collects the data, thereby displaying the corresponding data graph on the user interface. The monitoring system not only analyzes data but also plays a role in data viewing and storage. The correct execution of all systems is based on reasonable hardware, and the CPU used in the ZigBee wireless communication technology comes from the CC2530 single chip. The chip integrates SOC and supports the IEEE802.15.4 standard. The entire CPU also includes a powerful RF transceiver, programmable flash memory, and 8 KB of running memory. Its flash memory supports up to 256 KB. Because of its unique design, it also has personalized functions such as timing and customization [24]. The main structure of the sensor node is shown in Figure 6. Its components are temperature and humidity sensors, gas concentration sensors, water and electricity sensors, etc., as well as corresponding circuits and power supply devices. In the circuit of the temperature and humidity sensor, the coordinated work of CC2530 and CC2591 improves the working voltage and power of the node and further improves the stability of wireless transmission and increases the transmission range.

In view of the working environment of the sensor node, such as humidity and high and low temperature, the shell needs to use corrosion-resistant, waterproof, and dust-proof materials to protect the internal chips and circuits to ensure the normal operation of all nodes in the breeding environment. The detailed name of the gas concentration sensor is BGD-NH3 electrochemical sensor. The working principle of the sensor is to detect the concentration of the gas by reacting with the gas to be detected and generating a corresponding electrical signal. Its measurement accuracy is ±1%F.S, and its measurement range is 0~100 mg/L. The power consumption sensor mainly calculates the power consumption and transmits it via RS-485. Finally, the CC2530 uses the data frame command to read the relevant power consumption information. The water consumption sensor adopts a direct design, which reflects the real-time water consumption through the number of turns of the internal magnetic needle. The installation position of the magnetic needle will have a significant impact on the accuracy of the water consumption reading, so reasonable installation should be carried out according to the actual environment.

### 4.2. Experimental Results Based on Improved Genetic Algorithm

The genetic algorithm adopted in this article is different from the traditional genetic algorithm. The entire iterative process of the traditional genetic algorithm always uses a fixed crossover operator and mutation operator. The research method in the article is to combine the characteristics of a certain population in different time periods during the whole iterative process, so as to encourage the organisms in the population to make independent selection of hybridization operators and mutation operators. Through such a new genetic algorithm, we can effectively improve the accuracy of the algorithm and the reference value of the experimental structure. For a detailed analysis of the algorithm in the article, the main feature of the algorithm is the innovative introduction of two crossover operators, namely, directed crossover and random vector arithmetic crossover, which fully considers the universality and convergence in the calculation process, so as to avoid the premature occurrence of local optimal solutions in the algorithm and premature problems. Among them, the introduction of random vector arithmetic hybridization can ensure the fairness and stability of the algorithm during the entire iterative process. Therefore, at the beginning of the research, it is best to use random vector arithmetic hybridization. Because effective hybridization can improve the convergence of the overall algorithm, in the later stage of the research, the method of directional hybridization is adopted to promote the entire population to the most reasonable direction. After that, based on the three commonly used benchmark speed measurement functions, such as Rosenbrock, Rastrigin, and Griewank, we evaluate the performance of the adaptive genetic algorithm described above. When the number of iterations is set to 88 times, the results are shown in Tables 1–3.

The genetic algorithm used in the article is improved based on the multivariate continuous function. This algorithm is more stable in performance than traditional genetic algorithms, and its performance is smoother during the entire convergence process. At the same time, in the comparison of the two algorithms, the genetic algorithm used in the article has higher global optimization accuracy on the optimal optimization of complex multivariable continuous functions, and for the optimization of various objective functions, the algorithm performs better in terms of stability.

### 4.3. Temperature and Humidity Test Experiment Based on the Livestock Breeding Base Based on ZigBee Wireless Communication Network Sensor and the Above-Mentioned Improved Algorithm

In a certain breeding environment with universal reference value, perform relevant tests on the performance of the sensors used in reality. By using the new HOBOUX100-011 temperature and humidity recorder, the standard data of temperature and humidity in the breeding environment is selected. The recorder has built-in corresponding temperature and humidity sensors, and its effective temperature measurement range is -20°C~+70°C, and the test accuracy is ±0.21°C. The effective humidity measurement range is 5%~95%, and the test accuracy is ±2.5%RH. Before starting the test, debug the recorder correctly, and then connect the temperature and humidity sensor mentioned in Section 4.1. The factors tested in the experiment are temperature and humidity. A total of 9 times of temperature and humidity data were extracted before and after. Through the analysis of the data, the temperature and humidity were first tested indoors, and the measured values and actual values of indoor temperature and humidity can be compared as shown in Figure 7.

With reference to Figure 7, it can be seen that the temperature value collected from the environment differs from the actual value absolute value by 0.26°C, while the humidity value collected from the environment differs from the actual value absolute value by 0.25RH. It can be seen that the fluctuation of the value is within the normal usable range, so the results obtained by the experiment can meet the overall requirements, can ensure the normal operation of the system, and can be used in practical applications. Select a certain suburban livestock house with universal reference value to carry out the actual test of the relevant system. Through the operation of the system and the computer and the control of the relevant hardware equipment, the wireless and wired network communication and the monitoring function are correspondingly effectively tested. All sensors in the entire environment will be placed in the control cabinet. In the previous article, the stability and reliability of the system have been strictly verified. The entire system can accurately measure the effective adjustment of the accuracy of the new genetic algorithm to the sensor. During the entire experiment, the data storage and processing cycle are controlled to 12 s, which can more accurately measure the temperature and humidity changes in the environment, and the system will perform a parameter judgment and identification during this period. When the sensor is monitoring, the temperature comparison between using the improved genetic algorithm and not using it is shown in Figure 8.

It can be seen that the test data using the improved genetic algorithm has been greatly improved. When the temperature is tested, the average absolute value error without the algorithm is 0.29, but the average absolute value error of the improved genetic algorithm is only 0.034, and the error is relatively reduced by 88.28%, which is a great improvement.  Figure 9 shows the comparison of humidity with and without using improved genetic algorithm.

It can be seen that the test data using the improved genetic algorithm has been greatly improved. When the humidity is tested, the average absolute value error without algorithm is 0.19, but the average absolute value error of the improved genetic algorithm is only 0.03, and the error is relatively reduced by 84.21%, which is a great improvement.  Figure 10 shows the temperature and humidity absolute value error comparison with or without improved genetic algorithm.

The error of the improved genetic algorithm is extremely small, the temperature deviation is within 0.09, and the humidity deviation is within 0.08. The performance is obviously better, and it is extremely suitable for the temperature and humidity measurement and control of the livestock house.

## 5. Discussion

The breeding environment monitoring system developed and designed based on ZigBee wireless communication networking technology can effectively improve the problems of incomplete monitoring information of the breeding environment and low reference value. At the same time, it greatly reduces the manpower consumption and avoids errors caused by manual data recording. The monitoring system can perform multidimensional monitoring and analysis of a certain breeding environment, such as temperature and humidity, gas concentration, and water and electricity consumption in the current environment. The entire system can read, collect, summarize, process, and transmit data from each sensor completely autonomously and automatically. The relevant data is transmitted by the ZigBee wireless network to the upper computer monitoring system. This system can store, view, and analyze the received data. Through the application of the system in actual conditions, the results show that the system can indeed provide stable monitoring functions effectively, properly, and autonomously operate all kinds of information in the entire breeding environment, with low cost, less wiring, and high customization and scalability, so that it has extremely high application and promotion value. In an indoor breeding environment with universal reference value, adequate verification of the feasibility of the program is carried out. At the same time, the measurement of temperature and humidity in the outdoor breeding environment is also a complete program verification. During the entire control and monitoring process, a new genetic algorithm is used to strictly verify the control accuracy. Obtaining the corresponding data from the above experiments, visually display the data in the form of a line graph, which can reflect the performance change trend of the system during operation. Through the summary of experimental data, detailed data analysis is carried out to obtain the expected results.

## 6. Conclusions

In the experiment based on ZigBee wireless communication network sensor combined with improved genetic algorithm in the temperature and humidity test of the breeding farm, the data collection and monitoring system of the ZigBee network system is designed. As the temperature and humidity sensor to be used below, and use hybridization operator and mutation operator to improve the genetic algorithm, based on Rosenbrock, Rastrigin, and Griewank and other three commonly used benchmark speed measurement functions for algorithm testing, it is concluded that the algorithm is more stable in performance than the traditional genetic algorithm, and in the whole process of convergence, its performance is smoother and has higher global optimization accuracy. The temperature and humidity test experiment of the livestock breeding base is carried out again, and the average absolute value error without algorithm is 0.29 when the test temperature is tested, and the absolute value error under the improved algorithm is only 0.034, which is a relative decrease of 88.28%. In the humidity experiment, the average absolute value error without algorithm is 0.19, and the absolute value error under the improved algorithm is only 0.03, and the error is relatively reduced by 84.21%. And under the improved algorithm, the temperature deviation is within 0.09 and the humidity deviation is within 0.08, which has monitoring stability and has a good development prospect in the application of animal husbandry farms.

## Figures and Tables

**Figure 1:** The structure of the monitoring system for livestock breeding environment.

**Figure 2:** The overall hardware structure of the livestock breeding environment monitoring system.

**Figure 3:** Equipment structure of aquaculture environment parameter sensing concentrator.

**Figure 4:** Concept of trilateral positioning algorithm.

**Figure 5:** Link survival time estimation model.

**Figure 6:** Sensor acquisition node structure.

**Figure 7:** Indoor environment temperature and humidity comparison.

**Figure 8:** Comparison of temperature test results with and without this algorithm.

**Figure 9:** Comparison of humidity test results with and without this algorithm.

**Figure 10:** Comparison of the absolute value of the error of the temperature and humidity test results with and without the improved genetic algorithm.

**Table 1:** Rosenbrock function minimum optimization results.

Optimization	Average value	Standard deviation	The optimal value	Worst value	Time-consuming (seconds)
Traditional genetic algorithm	0.8301	1.1623	0.0138	5.0096	2.458
Gaussian mutation genetic algorithm	0.1427	0.1417	0.0024	0.5229	2.965
Improved genetic algorithm	4.48E-04	1.03E-03	6.19E-07	4.61E-03	3.146

**Table 2:** Optimization results of the minimum value of Rastrigin function.

Optimization	Average value	Standard deviation	The optimal value	Worst value	Time-consuming (seconds)
Traditional genetic algorithm	1.4122	1.2966	0.0152	5.3027	2.402
Gaussian mutation genetic algorithm	0.4198	0.4699	0.0056	1.8395	2.997
Improved genetic algorithm	2.45E-02	1.38E-01	1.34E-07	4.40E-03	3.983

**Table 3:** Minimum optimization results of Griewank function.

Optimization	Average value	Standard deviation	The optimal value	Worst value	Time-consuming (seconds)
Traditional genetic algorithm	0.9872	1.2853	0.0508	5.1266	2.451
Gaussian mutation genetic algorithm	0.0601	0.0499	3.86E-04	0.2012	3.697
Improved genetic algorithm	3.00E-03	4.00E-03	1.00E-06	1.11E-02	4.581

## Data Availability

No data were used to support this study.
